The article "Chaos in Cancer Tumor Growth Model with Commensurate and Incommensurate Fractional-Order Derivatives" was published in 2022. Journal: Comput Math Methods Med.

# Chaos in Cancer Tumor Growth Model with Commensurate and Incommensurate Fractional-Order Derivatives

**DOI:** 10.1155/2022/5227503

**Published:** 2022-05-20

**Authors:** Nadjette Debbouche, Adel Ouannas, Giuseppe Grassi, Abdul-Basset A. Al-Hussein, Fadhil Rahma Tahir, Khaled M. Saad, Hadi Jahanshahi, Ayman A. Aly

**Affiliations:** ^1^Department of Mathematics and Computer Science, University of Larbi Ben M'hidi, Oum El Bouaghi 04000, Algeria; ^2^Dipartimento Ingegneria Innovazione, Universita del Salento, 73100 Lecce, Italy; ^3^Electrical Engineering Department, College of Engineering, University of Basrah, Basrah, Iraq; ^4^Department of Mathematics, Faculty of Applied Science, Taiz University, Taiz, Yemen; ^5^Department of Mechanical Engineering, University of Manitoba, Winnipeg, MB R3T 5V6, Canada; ^6^Department of Mechanical Engineering, College of Engineering, Taif University, P.O.Box 11099, Taif 21944, Saudi Arabia

## Abstract

Analyzing the dynamics of tumor-immune systems can play an important role in the fight against cancer, since it can foster the development of more effective medical treatments. This paper was aimed at making a contribution to the study of tumor-immune dynamics by presenting a new model of cancer growth based on fractional-order differential equations. By investigating the system dynamics, the manuscript highlights the chaotic behaviors of the proposed cancer model for both the commensurate and the incommensurate cases. Bifurcation diagrams, the Lyapunov exponents, and phase plots confirm the effectiveness of the conceived approach. Finally, some considerations regarding the biological meaning of the obtained results are reported through the manuscript.

## 1. Introduction

In the last fifty years, great research efforts and economic resources have been directed to win the fight against cancer. In order to tackle the problem, one of the key issues is to active and control the immune system in its competition against neoplastic cells [1]. To this purpose, the study of tumor-immune dynamics can play a role of paramount importance, given that the mathematical modeling of cancer growth is considered one of the useful tools for the development of effective medical treatments [2, 3]. Over the years, the study of the tumor-immune dynamics has led to the discovery of remarkable phenomena, including the presence of chaos in the system dynamics. By considering integer-order dynamical systems (i.e., biological systems described by integer-order differential equations), in [4], a simple chaotic model of three competing cell populations (host, immune, and tumor cells) is introduced. Topological analysis and computing observability coefficients are illustrated, with the aim to suggest new trends in understanding the interactions of some tumor cells [4]. The authors of reference [5] have suggested a suitable model for the tumor growth, i.e., a discrete-time system capable of exhibiting periodic and chaotic behaviors. The model, which is validated through experimental data, can explain a number of biologically observed tumor states and dynamics [5]. Another interesting model of tumor growth is proposed in [6], based on the interactions among tumor cells, healthy tissue cells, and activated immune system cells. The study, besides analyzing the stability of the system equilibria, highlights the presence of chaotic behaviors in the system dynamics [6]. Referring to biological systems, it should be noted that the behavior of most of these systems has memory or aftereffects [7]. Moreover, biological systems are usually characterized by hereditary properties and nonlocal distributed behaviors. As a consequence, the modeling of these systems by fractional-order differential equations has more advantages than integer-order modeling, in which such effects are neglected [7]. This explains why fractional calculus has recently emerged as a valuable tool for describing a number of dynamic phenomena in biological systems [8]. Regarding tumor-immune dynamics, in [7], a fractional-order model with two immune effectors interacting with the cancer cells is introduced. The conditions that guarantee the stability of the equilibrium points in the considered fractional cancer model are discussed in details [7]. In [9], a mathematical model of cancer chemotherapy effect involving the Caputo fractional derived is presented. In [10], a fractional model of cancer-immune system with Caputo and Caputo-Fabrizio derivatives is investigated. In particular, after examining the stability of the system with singular kernel, the existence and uniqueness of the numerical solution is discussed [10]. In [11], a novel fractional model for a tumor-immune surveillance mechanism is introduced. The approach, besides analyzing the interactions between various tumor cell populations and immune systems, provides an optimal control strategy for investigating the effects of chemotherapy treatments [11]. While references [9–11] have mainly investigated the properties of the mathematical model under consideration, a number of papers have recently focused on the presence of chaos in fractional-order cancer models [12–16]. For example, reference [12] has been one of the first papers to investigate the presence of chaos in fractional-order cancer models. In particular, in [12], the authors have developed a fractional chaotic dynamical model of cancer growth, which includes the interactions between healthy tissue cells, tumor cells, and activated immune system cells. The existence of chaos for the commensurate and incommensurate fractional cancer systems (with order less than 3) is investigated [12]. In [13], a fractional discrete version of a tumor-immune system interaction is analyzed. This model, derived via a discretization process where conformable fractional derivatives are taken into account, exhibits bifurcations and chaotic behaviors [13]. In [14], a study of tumor and effector cells through fractional tumor-immune dynamical model is conducted. By using the Mittag-Leffler law, the paper highlights the existence of chaos in the considered fractional tumor-immune model for cancer treatment [14]. In [15], three-dimensional cancer models that include the interactions between tumor cells, healthy tissue cells, and activated immune system cells are considered. The systems, which are described via Liouville-Caputo, Caputo-Fabrizio, Atangana-Baleanu, and fractional conformable derivatives, show a number of chaotic attractors with symmetric scrolls, depending on the type of the selected derivative [15]. In [16], a cancer model involving the new fractional derivative with the Mittag-Leffler kernel in Liouville-Caputo sense is investigated. A large variety of chaotic attractors is shown, along with the uniqueness and existence of the solutions in the fractional cancer system [16]. Based on these considerations, this paper was aimed at making a contribution to the study of tumor-immune dynamics by presenting a new model of cancer growth based on fractional-order differential equations. By investigating the system dynamics, the manuscript highlights the chaotic behaviors of the proposed cancer model for both the commensurate and the incommensurate cases. Moreover, some considerations regarding the biological meaning of the obtained results are reported. The paper is organized as follows. In Section 2, a novel fractional-order cancer model based on the Caputo derivative is presented. Moreover, a stability analysis of the system equilibria is conducted. In Section 3, by varying the value of the fractional order as well as the values of the system parameters, the dynamics of the commensurate fractional cancer model are analyzed via bifurcation diagrams, the Lyapunov exponents, and phase plots. When the order of the derivative goes beyond the threshold value, *q* > 0.96, chaotic behaviors are found, indicating that the number of the tumor cells of the healthy host cells and of the effector cells becomes unpredictable. Finally, in Section 4, the dynamics of the incommensurate fractional cancer model are analyzed in details by varying the value of the fractional order in each system equation. Simulation results reported through the manuscript highlight that the proposed approach can explain many biologically observed tumor states (including stable, periodic, and chaotic behaviors), indicating that under some conditions the interactions between tumor cells, healthy tissue cells, and activated immune system cells could lead to invasive tumor growth.

The article "Chaos in Cancer Tumor Growth Model with Commensurate and Incommensurate Fractional-Order Derivatives" was published in 2022. Journal: Comput Math Methods Med.

## 2. Fractional-Order Cancer Model and Its Equilibrium Points

A three-dimensional integer-order cancer growth model has been studied in [6]. Its dynamic equations are described by [17]:

(1) $$\begin{array}{c} \left\{\begin{array}{c} \dot{x}=ax\left(1-y\right)\left(1+z\right)-x^{2}y,\\ \dot{y}=by\left(1-z\right)\left(1+x\right)-y^{2}z,\\ \dot{z}=cz\left(1-x\right)\left(1+y\right)-z^{2}x, \end{array}\right. \end{array}$$

where *x*(*t*) denotes the number of tumor cells at time *t*, *y*(*t*) is the number of healthy host cells at time *t*, and *z*(*t*) refers to the number of effector immune cells at time *t* in the single tumor-site compartment. Here, the parameters *a*, *b*, and *c* are positive real numbers representing the growth rates of populations of *x*(*t*), *y*(*t*), and *z*(t) (see [6]). Specifically, the parameter *a* represents the growth rate of the tumor cells (measured in sec-1), the parameter *b* is the growth rate of the healthy host cells (measured in sec-1), whereas *c* represents the growth rate of the effector immune cells (measured in sec-1). Generally, the model parameters are chosen such that the system dynamic analogies with clinical evidences reported in literatures [4, 18], where depending on control parameter values and initial conditions, the considered biological cancerous system should also approach different states [19]: stationary equilibrium state where any changes are damped, stable periodic process (a limit cycle), and state of instability with chaotic behavior. As shown in [6], particular values of these growth rates lead to make the behavior of system (1) chaotic. To this purpose, the chaotic attractor of system (1) for parameters *a* = 0.7455, *b* = 0.7367, and *c* = 0.5619 and initial conditions (*x*_0_, *y*_0_, *z*_0_) = (0.4,0.5,0.5) is shown in Figure 1.

Herein, the fractional version of system (1) is considered. Namely, the dynamics of the proposed fractional-order cancer model (FOCM) are described by

(2) $$\begin{array}{c} \left\{\begin{array}{c} D_{t}^{q_{1}}x=ax\left(1-y\right)\left(1+z\right)-x^{2}y,\\ D_{t}^{q_{2}}y=by\left(1-z\right)\left(1+x\right)-y^{2}z,\\ D_{t}^{q_{3}}z=cz\left(1-x\right)\left(1+y\right)-z^{2}x, \end{array}\right. \end{array}$$

where *D*^*q*^ is *q*-order Caputo differential operator, 0 < *q*_*i*_ ≤ 1(*i* = 1, 2, 3) are the derivative orders of the state variables *x*, *y*, and *z* (see appendix A). The fractional-order system (2) is called as commensurate if *q*_1_ = *q*_2_ = *q*_3_ and incommensurate otherwise.

The article "Chaos in Cancer Tumor Growth Model with Commensurate and Incommensurate Fractional-Order Derivatives" was published in 2022. Journal: Comput Math Methods Med.

Using the definitions (Equations (B.3) and (B.4)) in Appendix B, then the numerical solution of the FOCM can be given as in (3) with parameters defined in (4) and (5), where *l* = 1, 2, 3 and *i* = 1, 2, 3.

(3) $$\begin{array}{c} \left\{\begin{array}{c} x_{n+1}=x_{0}+\frac{h^{q_{1}}}{\Gamma \left(q_{x}+2\right)}\left[ax_{1+n}^{p}\left(1-y_{1+n}^{p}\right)\left(1+z_{1+n}^{p}\right)-{\left(x_{1+n}^{p}\right)}^{2}y_{1+n}^{p}\right]\\ +\frac{h^{q_{1}}}{\Gamma \left(q_{x}+2\right)}\overset{n}{\underset{j=0}{\sum }}\left[\eta_{1,j,n+1}\left(ax_{j}\left(1-y_{j}\right)\left(1+z_{j}\right)-x_{j}^{2}y_{j}\right)\right],\\ y_{n+1}=y_{0}+\frac{h^{q_{2}}}{\Gamma \left(q_{y}+2\right)}\left[by_{1+n}^{p}\left(1-z_{1+n}^{p}\right)\left(1+x_{1+n}^{p}\right)-{\left(y_{1+n}^{p}\right)}^{2}z_{1+n}^{p}\right]\\ +\frac{h^{q_{2}}}{\Gamma \left(q_{y}+2\right)}\overset{n}{\underset{j=0}{\sum }}\left[\eta_{2,j,n+1}\left(by_{j}\left(1-z_{j}\right)\left(1+x_{j}\right)-y_{j}^{2}z_{j}\right)\right],\\ z_{n+1}=z_{0}+\frac{h^{q_{3}}}{\Gamma \left(q_{z}+2\right)}\left[cz_{1+n}^{p}\left(1-x_{1+n}^{p}\right)\left(1+y_{1+n}^{p}\right)-{\left(z_{1+n}^{p}\right)}^{2}x_{1+n}^{p}\right]\\ +\frac{h^{q_{3}}}{\Gamma \left(q_{z}+2\right)}\overset{n}{\underset{j=0}{\sum }}\left[\eta_{3,j,n+1}\left(cz_{j}\left(1-x_{j}\right)\left(1+y_{j}\right)-z_{j}^{2}x_{j}\right)\right], \end{array}\right. \end{array}$$

(4) $$\begin{array}{c} \left\{\begin{array}{c} x_{n+1}^{p}=x_{0}+\frac{1}{\Gamma \left(q_{1}+2\right)}\overset{n}{\underset{j=0}{\sum }}\omega_{1,j,n+1}\left(ax_{j}\left(1-y_{j}\right)\left(1+z_{j}\right)-x_{j}^{2}y_{j}\right),\\ y_{n+1}^{p}=y_{0}+\frac{1}{\Gamma \left(q_{2}+2\right)}\overset{n}{\underset{j=0}{\sum }}\omega_{2,j,n+1}\left(by_{j}\left(1-z_{j}\right)\left(1+x_{j}\right)-y_{j}^{2}z_{j}\right),\\ z_{n+1}^{p}=z_{0}+\frac{1}{\Gamma \left(q_{3}+2\right)}\overset{n}{\underset{j=0}{\sum }}\omega_{3,j,n+1}\left(cz_{j}\left(1-x_{j}\right)\left(1+y_{j}\right)-z_{j}^{2}x_{j}\right), \end{array}\right. \end{array}$$

(5) $$\begin{array}{c} \left\{\begin{array}{c} \eta_{l,j,n+1}=\left\{\begin{array}{cc} n^{q_{i}+1}-\left(n-q_{i}\right){\left(n+1\right)}^{q_{i}+1}, & j=0,\\ {\left(n-j+2\right)}^{q_{i}+1}+{\left(n-j\right)}^{q_{i}+1}-2{\left(n-j+1\right)}^{q_{i}+1}, & 1\leq j\leq n,\\ 1, & j=n+1, \end{array}\right.\\ \omega_{l,j,n+1}=\frac{h^{q_{i}}}{q_{i}}\left({\left(n-j+1\right)}^{q_{i}}-{\left(n-j\right)}^{q_{i}}\right),0\leq l\leq n. \end{array}\right. \end{array}$$

Note that system (2) has five equilibrium points [6], four of them are obtained analytically and can be described as follows:

1. *E*_0_ = (0, 0, 0),
2. *E*_1_ = (0, −1, (*b*/*b* − 1)), if *b* ≠ 1
3. *E*_2_ = ((*c*/*c* − 1), 0, −1), if *c* ≠ 1
4. *E*_3_ = (−1, (*a*/*a* − 1), 0), if *a* ≠ 0

The last equilibrium *E*_4_ corresponding to the case (*x*, *y*, *z*) ≠ (0, 0, 0) does not possess an analytical expression. It could be obtained by intersecting the three surfaces corresponding to the following equations:

(6) $$\begin{array}{c} \left\{\begin{array}{c} ax\left(1-y\right)\left(1+z\right)-x^{2}y=0,\\ by\left(1-z\right)\left(1+x\right)-y^{2}z=0,\\ cz\left(1-x\right)\left(1+y\right)-z^{2}x=0. \end{array}\right. \end{array}$$

By taking the system parameters *a* = 0.7455, *b* = 0.7367, and *c* = 0.5619, the fixed points become *E*_0_ = (0, 0, 0), *E*_1_ = (0, −1, −2.7979), *E*_2_ = (−1.28,0, −1), *E*_3_ = (−1, −2.9293,0), and the fourth equilibrium point found as *E*_4_ = (0.5961, 0.6718,0.6364), as shown in Figure 2.

The article "Chaos in Cancer Tumor Growth Model with Commensurate and Incommensurate Fractional-Order Derivatives" was published in 2022. Journal: Comput Math Methods Med.

Note that the fixed points *E*_1_, *E*_2_, and *E*_3_ have negative coordinates, indicating that the dynamics cannot take place since it is not possible to define negative populations in system (2). The fixed point *E*_0_, which corresponds to a situation where there is no cell at all, is unstable, since its eigenvalues are given by (0.5619,0.7367, and 0.7455). The fixed point *E*_4_, which is associated with the coexistence of the three different types of cells, represents a saddle-focus equilibrium, since its eigenvalues are given by (0.0712 ± 1.0922*i*, 1.3498).

## 3. Dynamics of the Commensurate Fractional-Order Cancer Model

In this section, the dynamics of the proposed commensurate fractional-order cancer model (2) are studied by varying the fractional-order *q* and the system parameters *a*, *b*, and *c*. The bifurcation diagrams, Lyapunov exponents, time behaviors, and phase plots are illustrated to investigate the system dynamics in detail. Moreover, some considerations regarding the biological meaning of the obtained results are reported.

### 3.1. Analysis of the System Dynamics by Varying the Fractional-Order *q*

The study of the stability of the equilibria is important to understand the system dynamics in the proposed cancer model. Herein, analytical and numerical analyses are conducted to determine the behavior of the system trajectories when the value of the fractional order is properly varied. To this purpose, a theorem proved in reference [20] is now exploited.

**Theorem 1 .**

Given the fractional system (2), a necessary condition to have a chaotic attractor around the equilibrium point E_4_ is that the eigenvalues *λ*_i_ of its Jacobian matrix satisfy the condition [20]:

(7) $$\begin{array}{c} \arg\left(\lambda_{i}\right)>q\pi /2,0<q<1, \end{array}$$

By taking the fractional system (2) with parameters *a* = 0.7455, *b* = 0.7367, and *c* = 0.5619, the eigenvalues *λ*_*i*_, *i* = 1, 2, 3 of the Jacobian matrix are evaluated at the equilibrium point *E*_4_ are given by (0.0712 ± 1.0922*i*, −1.3498). By considering that the application of Theorem 1 to the equilibrium *E*_4_ gives

(8) $$\begin{array}{c} \arg\left(0.0712\pm 1.0922i\right)*2/pi\approx 0.9576, \end{array}$$

it follows that a necessary condition to have a chaotic attractor in the fractional system (2) is to satisfy the condition *q* > 0.96.

The article "Chaos in Cancer Tumor Growth Model with Commensurate and Incommensurate Fractional-Order Derivatives" was published in 2022. Journal: Comput Math Methods Med.

In order to investigate the system dynamics and numerically search for proper values of the fractional-order*q* which is able to generate chaotic behaviors, the bifurcation diagram is plotted in Figure 3 for *q* ∈ (0.94,1) and initial conditions (*x*_0_, *y*_0_, *z*_0_) = (0.4,0.5,0.5).

From the bifurcation diagram, it can be seen that system (2) is asymptotically stable when *q* < 0.96, whereas a number of periodic windows appear for *q* ∈ (0.96,0.99). Moreover the FOCM (2) exhibits chaotic behavior for *q* ∈ (0.99,1) as confirmed by the positive values of the maximum Lyapunov exponents (see Figure 4). From the biological point of view, this behavior can be explained as follows. When *q* < 1, the system become fractional and, consequently, memory effects and hereditary properties appear in the modeling of the system dynamics. When these effects are not so strong (i.e., 0.99 < *q* < 1), the system dynamics undertake chaotic behaviors. On the other hand, when these effects become stronger (i.e., *q* < 0.96), they overwhelm the system dynamics, which undertake stable behaviors.

By varying the value of the fractional-order *q*, Figure 5 shows the time behaviors of the three state variables: *x*(*t*), *y*(*t*), and *z*(*t*) (in red, blue, and green color, respectively) along with the corresponding phase portraits in the *x*-*y* plan, for the system parameters *a* = 0.7455, *b* = 0.7367, and *c* = 0.5619 and initial conditions (*x*_0_, *y*_0_, *z*_0_) = (0.4,0.5,0.5). When *q* = 0.95, it can be observed that the FOCM (2) is asymptotically stable and the system trajectories converge to the equilibrium point *E*_4_ (Figure 5(a)). When *q* = 0.962, the system loses its stability and a scroll begins to appear around the point *E*_4_ (Figure 5(b)). By increasing the values of *q*, periodic attractors appear for *q* = 0.97 and *q* = 0.98 (Figures 5(c) and 5(d)). When *q* = 0.995, the fractional cancer model (2) exhibits a chaotic attractor (Figure 5(e)), which is similar to that one obtained for the integer-order case (Figure 5(f)).

The article "Chaos in Cancer Tumor Growth Model with Commensurate and Incommensurate Fractional-Order Derivatives" was published in 2022. Journal: Comput Math Methods Med.

A projection in the 3D space of the chaotic attractor generated by the proposed fractional-order cancer model is plotted in Figure 6 for *q* = 0.995. The conducted analyses clearly indicate that, in order to get chaos, the theoretical condition expressed by Theorem 1 is numerically fulfilled when *q* = 0.995. From this results it can be concluded that, when the value of the fractional order decreases, the system becomes stable, indicating that the number of the tumor cells, of the healthy cells, and of the effector cells asymptotically converges to the equilibrium point. On the other hand, when the order of the derivative increases and goes beyond the value of *q* > 0.96, the dynamics of the proposed FOCM turn to be chaotic, indicating that the number of tumor cells, of the healthy host cells, and of the effector cells becomes unpredictable.

### 3.2. Analysis of the System Dynamics by Varying the Parameters *a*, *b*, and *c*

Herein, the analysis of the system dynamics is conducted by taking the fractional-order *q* = 0.99 and the initial conditions (*x*_0_, *y*_0_, *z*_0_) = (0.4,0.5,0.5) and by varying the parameters *a*, *b*, and *c*. At first, the parameters *a* and *c* are selected as *a* = 0.7455 and *c* = 0.5619, whereas the parameter *b* is varied in the interval (0, 1). Note that the parameter *b* is related to the growth rate of host cells. Since the best strategy to face the cancer dynamics, from the biological point of view, is to act on the healthy host cells [4], herein the parameter *b* is varied, with the aim to investigate the behavior of the proposed cancer model. The bifurcation diagrams of the three state variables *x*(*t*), *y*(*t*), and *z*(*t*) of the FOCM (2) are shown in Figure 7, where *b* is the bifurcation parameter.

By varying the value of the parameter *b*, Figure 8 shows the time behaviors of the three state variables: *x*(*t*), *y*(*t*), and *z*(*t*) (in red, blue, and green color, respectively) along with the corresponding phase portraits in the *x*-*y* plan for the system parameters *a* = 0.7455 and *c* = 0.5619 and initial conditions (*x*_0_, *y*_0_, *z*_0_) = (0.4,0.5,0.5). When *b* = 0.28, it can be observed that the FOCM (2) is asymptotically stable and the system trajectories converge to the equilibrium point *E*_4_ (Figure 8(a)). When the parameter *b* increases, a periodic route to chaos appears in the range *b* ∈ (0.30,0.5). In this range of parameter *b*, the system exhibits limit cycles of different periods (see Figures 8(b) and 8(c)). Then, a chaotic attractor appears at *b* = 0.53 (see Figure 8(d)) and the system exhibits a chaotic behavior for *b* ∈ (0.53,1).

The article "Chaos in Cancer Tumor Growth Model with Commensurate and Incommensurate Fractional-Order Derivatives" was published in 2022. Journal: Comput Math Methods Med.

Now, the parameter *b* is fixed at the value *b* = 0.7367, whereas the parameter *a*, which represents the growth rate of the tumor cells, is varied in the interval (0, 1). The corresponding bifurcation diagram for the three state variables *x*(*t*), *y*(*t*), and *z*(*t*) is plotted in Figure 9(a). Similarly, by fixing the value *b* = 0.7367, the parameter *c* (i.e, the growth rate of the effector cells) is varied in the interval (0, 1). The corresponding bifurcation diagram for the three state variables *x*(*t*), *y*(*t*), and *z*(*t*) is plotted in Figure 9(b). By analyzing the two bifurcation diagrams, it can be argued that the FOCM (2) loses its stability when the values of the parameters *a* and *c* are increased. Moreover, chaotic behaviors appear in the FOCM (2) when *a* ∈ (0.5,1) and *c* ∈ (0.35,1).

Regarding the biological meaning of these results, it should be noted that, for low values of the growth rates, the FOCM (2) has a stable equilibrium point. On the other hand, when the growth rates increase, the system loses its stability. At this stage, the tumor is ready to become invasive and even malignant [5]. With the further increase of the growth rates, the chaotic attractor of the tumor appears, being this higher tumor burden complicated by the presence of several periodic and chaotic dynamics. This is similar to what happens when parameter *b* increases in Figure 8. On the other hand, when the growth rates decrease, the attractor corresponding to high tumor burden disappears. This is similar to what happens when *a*, *b*, and *c* decrease in Figures 7 and 9. These results can help the doctors for controlling the tumor burden, thus giving suggestions regarding the medical treatments.

### 3.3. Comparison between the Dynamics of Integer-Order and Commensurate Fractional-Order Cancer Models

Now, comparisons between the dynamics of integer-order and commensurate fractional-order cancer models are carried out. The time behaviors of the state variable *x*(*t*) (representing the tumor population) are plotted in Figure 10 by selecting *q* = 0.90, *q* = 0.95, *q* = 0.99, and *q* = 1 and by taking different values of the system parameters *a*, *b*, and *c* ranges. It can be observed that for smaller values of the parameter *a* (Figure 10(a)), of the parameter *b* (Figure 10(c)), and of the parameter *c* (Figure 10(e)), the commensurate fractional derivatives damp the oscillation behavior. Consequently, the three states of tumor, host, and effector cells approach faster the equilibrium point, indicating that the commensurate fractional derivatives enlarge the region of stability. When the values of the parameters *a*, *b*, and *c* increase, the system is stable for small values of the fractional orders (i.e., *q* = 0.90 and *q* = 0.95). Namely, by looking at Figures 10(b), 10(d), and 10(e), it can be observed that the system trajectories tend to the equilibrium point for *q* = 0.90 and *q* = 0.95. On the other hand, chaotic oscillations with different amplitudes appear when for *q* = 0.995 and *q* = 1. Note that the amplitude of the chaotic oscillation reaches the maximum value for the integer-order case (*q* = 1).

The article "Chaos in Cancer Tumor Growth Model with Commensurate and Incommensurate Fractional-Order Derivatives" was published in 2022. Journal: Comput Math Methods Med.

## 4. Dynamics of the Incommensurate Fractional-Order Cancer Model

This section analyzes the dynamics of the incommensurate FOCM (2) by taking the parameters *a* = 0.7455, *b* = 0.7367, and *c* = 0.5619 and initial conditions (*x*_0_, *y*_0_, *z*_0_) = (0.4,0.5,0.5) and by selecting different values of the fractional-orders *q*_1_, *q*_2_, and *q*_3_. At first, the bifurcation diagrams of the variable *x*(*t*) are plotted in Figure 11(a) for three cases: *q*_1_ ∈ (0.6,1) and *q*_2_ = *q*_3_ = 1; *q*_2_ ∈ (0.6,1) and *q*_1_ = *q*_3_ = 1; *q*_3_ ∈ (0.6,1) and *q*_1_ = *q*_2_ = 1. From Figure 11(a), it can be seen that the equilibrium point is asymptotically stable when *q*_1_ < 0.75, *q*_2_ < 0.74, and *q*_3_ < 0.74. When the values of *q* increase, periodic windows appear for *q*_1_ ∈ (0.75,0.86), *q*_2_ ∈ (0.74,0.85), and *q*_3_ ∈ (0.74,0.85), whereas chaotic behaviors are exhibited for *q*_1_ ∈ (0.86,1), *q*_2_ ∈ (0.85,1), and *q*_3_ ∈ (0.85,1). The existence of positive Lyapunov exponents is confirmed by the plot as a function of the fractional-order *q*, as shown in Figure 11(b). Namely, from Figure 11(b), it can be seen that the fractional cancer system (2) is chaotic for *q*_1_ ∈ (0.86,1), *q*_2_ ∈ (0.85,1), and *q*_3_ ∈ (0.85,1). Note that the maximum value of the variable *x*(*t*) is obtained by varying *q*_3_ (see Figure 11(a)).

Figure 12 shows the time behaviors of the three state variables *x*(*t*), *y*(*t*), and *z*(*t*) (in red, blue, and green color, respectively) along with the corresponding phase portraits in the *x*-*y* plan, for the system parameters *a* = 0.7455, *b* = 0.7367, and *c* = 0.5619 and initial conditions (*x*_0_, *y*_0_, *z*_0_) = (0.4,0.5,0.5). By taking different values of the fractional-order *q*_1_, *q*_2_, and *q*_3_ in the incommensurate FOCM (2), some chaotic attractors appear. For example, Figure 12(a) plots the chaotic attractor obtained for *q*_1_ = 0.999 and *q*_2_ = *q*_3_ = 1, whereas Figures 12(b) and 12(c) illustrate the chaotic attractors obtained for *q*_2_ = 0.999*q*_1_ = *q*_3_ = 1 and for *q*_3_ = 0.999, *q*_1_ = *q*_2_ = 1, respectively. By looking at the time behaviors of the state variables, it can be noticed that the maximum amplitudes of the trajectories change from one plot to the other when the incommensurate orders are varied. Specifically, the population of the healthy host cells (i.e., the state variable *y*(*t*)) is the largest when *q*_1_ = 0.999 (see Figure 12(a)), the population of the effector immune cells (i.e., the state variable *z*(*t*)) is the largest when *q*_2_ = 0.999 (see Figure 12(b)), whereas the population of the tumor cells (i.e., the state variable *x*(*t*)) is the largest when *q*_3_ = 0.999 (see Figure 12(c)).

The article "Chaos in Cancer Tumor Growth Model with Commensurate and Incommensurate Fractional-Order Derivatives" was published in 2022. Journal: Comput Math Methods Med.

Now, by fixing the system parameters *a* = 0.7455 and *c* = 0.5619, the bifurcation diagrams for the variable *x*(*t*) as a function of the parameter *b* are derived for three cases: *q*_1_ = 0.999, *q*_2_ = *q*_3_ = 1; *q*_2_ = 0.999, *q*_1_ = *q*_3_ = 1; and *q*_3_ = 0.999, *q*_1_ = *q*_2_ = 1 (see Figure 13). It can be noticed that the incommensurate system (2) exhibits chaos in all the three cases when *b* ∈ (0.38,1).

Figure 14 presents the chaotic attractors of the incommensurate FOCM (2) in 3D projection by taking the parameter *b* = 0.38 for: (a) *q*_1_ = 0.999, *q*_2_ = *q*_3_ = 1; (b) *q*_2_ = 0.999, *q*_1_ = *q*_3_ = 1; and (c) *q*_3_ = 0.999, *q*_1_ = *q*_2_ = 1. By comparing this chaotic range with the range that has been obtained in Section 3 (see Figures 7 and 8), it can be observed that the incommensurate fractional derivatives enlarge the chaotic range of the solution. From the biological point of view, it can be deduced that, when the growth rate decreases, the attractor corresponding to the high tumor burden disappears. This is in accordance with the results in Figure 13, since when *b* decreases the system dynamics go towards stable behaviors.

Now, comparisons between the dynamics of integer-order and incommensurate fractional-order cancer models are carried out. The time behaviors of the state variable *x*(*t*) (representing the tumor population) are plotted in Figure 15 by selecting different values of the fractional-orders *q*_1_, *q*_2_, and *q*_3_, when the parameter *b* assumes the two values *b* = 0.1 (corresponding to the stable range) and *b* = 0.5 (corresponding to the chaotic range). It can be observed that for *b* = 0.1 (see Figures 15(a), 15(c), and 15(e)), the incommensurate fractional derivatives damp the oscillation behavior. Consequently, the three states of tumor, host, and effector cells approach faster the equilibrium point, indicating that the incommensurate fractional derivatives enlarge the region of stability. When the parameter *b* assumes the value *b* = 0.5, the system is stable for small values of the fractional orders (i.e., *q*_1_, *q*_2_, *q*_3_ = 0.60, *q*_1_, *q*_2_, *q*_3_ = 0.80). Namely, by looking at Figures 15(b), 15(d), and 15(e), it can be observed that the system trajectories tend to the equilibrium point for *q*_1_, *q*_2_, *q*_3_ = 0.60 and *q*_1_, *q*_2_, *q*_3_ = 0.80. On the other hand, chaotic oscillations with different amplitudes appear when *q*_1_, *q*_2_, *q*_3_ = 0.995 and *q*_1_, *q*_2_, *q*_3_ = 1. Note that the amplitude of the chaotic oscillation reaches the maximum value for the integer-order case (*q*_1_, *q*_2_, *q*_3_ = 1). The motivation of the manuscript is to provide a complete study of tumor-immune dynamics by presenting a new model of cancer growth. In order to explain the physical meaning of introducing the fractional-order into the model, it is worth noting that biological systems are characterized by memory or aftereffects, hereditary properties, and nonlocal distributed behaviors [7]. Since these features are neglected in integer-order modeling, this has motivated the use of fractional calculus as a tool for accurately describing dynamic phenomena in tumor-immune systems. The main advantage of the results in this paper, compared with others published in the literature, is that our approach represents an exhaustive study of tumor-immune dynamics, since it includes the bifurcation diagrams, Lyapunov exponents, and phase plots for both the commensurate and the incommensurate cases. No paper published in the literature so far (to the best of the authors' knowledge) includes such a complete analysis of the fractional chaotic dynamics of tumor-immune systems [12–16].

The article "Chaos in Cancer Tumor Growth Model with Commensurate and Incommensurate Fractional-Order Derivatives" was published in 2022. Journal: Comput Math Methods Med.

## 5. Conclusion

This paper has made a contribution to the study of tumor-immune dynamics by presenting a new model of cancer growth based on fractional-order differential equations. By investigating the system dynamics, the manuscript has highlighted the chaotic behaviors of the proposed cancer model for both the commensurate and the incommensurate cases. In particular, by using the bifurcation diagrams, Lyapunov exponents, phase plots, and a necessary condition to get chaos, the paper has shown that, when the order of the derivative goes beyond the threshold value *q* > 0.96, different chaotic behaviors are found, indicating that the number of the tumor cells, of the healthy host cells, and the effector cells becomes unpredictable. Finally, simulation results reported through the manuscript have highlighted that the proposed approach can explain many biologically observed tumor states, including stable, periodic, and chaotic behaviors. Regarding open research problems, an important issue is related to the development of control techniques for suppressing chaos in fractional-order biological systems. Our future plan is to work on this issue, since we believe that controlling chaos in fractional tumor-immune systems might help biologists in the fight against cancer.

The article "Chaos in Cancer Tumor Growth Model with Commensurate and Incommensurate Fractional-Order Derivatives" was published in 2022. Journal: Comput Math Methods Med.

## Figures and Tables

**Figure 1:** Chaotic attractor of system (1) for system parameters *a* = 0.7455, *b* = 0.7367, and *c* = 0.5619 and initial conditions (*x*_0_, *y*_0_, *z*_0_) = (0.4,0.5,0.5).

**Figure 2:** Equilibrium point *E*_4_ obtained by intersecting the three surfaces corresponding to Equation (6).

**Figure 3:** Bifurcation diagram of commensurate FOCM for *q* ∈ (0.94,1) with parameters *a* = 0.7455, *b* = 0.7367, and *c* = 0.5619 and initial conditions (*x*_0_, *y*_0_, *z*_0_) = (0.4,0.5,0.5).

**Figure 4:** The maximum Lyapunov exponent of the commensurate FOCM (2) for *q* ∈ (0.99,1) with parameters *a* = 0.7455, *b* = 0.7367, and *c* = 0.5619 and initial conditions (*x*_0_, *y*_0_, *z*_0_) = (0.4,0.5,0.5).

**Figure 5:** Time behaviors of the three state variables *x*(*t*), *y*(*t*), and *z*(*t*) (in red, blue, and green color, respectively) along with the corresponding phase portraits in the *x*-*y* plan, when *a* = 0.7455, *b* = 0.7367, and *c* = 0.5619 and initial conditions (*x*_0_, *y*_0_, *z*_0_) = (0.4,0.5,0.5) for: (a) *q* = 0.95, (b) *q* = 0.962, (c) *q* = 0.97, (d) *q* = 0.98, (e) *q* = 0.995, and (f) *q* = 1.

**Figure 6:** Projection in the 3D space of the chaotic attractor of commensurate FOCM for *q* = 0.995 when *a* = 0.7455, *b* = 0.7367, and *c* = 0.5619 and initial conditions (*x*_0_, *y*_0_, *z*_0_) = (0.4,0.5,0.5).

**Figure 7:** (a) Bifurcation diagrams of commensurate FOCM for *q* = 0.99, *a* = 0.7455, *c* = 0.5619, and (*x*_0_, *y*_0_, *z*_0_) = (0.4,0.5,0.5) by varying parameter *b* ∈ (0, 1) for: (a) *x*(*t*) state variable, (b) *y*(*t*) state variable, and (c) *z*(*t*) state variable.

**Figure 8:** Time behaviors of the three state variables: *x*(*t*), *y*(*t*), and *z*(*t*) (in red, blue, and green color, respectively) along with the corresponding phase portraits in the *x*-*y* plan when *q* = 0.99, *a* = 0.7455, *c* = 0.5619, and (*x*_0_, *y*_0_, *z*_0_) = (0.4,0.5,0.5) for: (a) *b* = 0.28, (b) *b* = 0.38, (c) *b* = 0.45, and (d) *b* = 0.53.

**Figure 9:** Bifurcation diagrams of the variables: *x*(*t*), *y*(*t*), and *z*(*t*) (in red, blue, and green color, respectively) of the commensurate FOCM (2) with *q* = 0.99, *b* = 0.7367, and (*x*_0_, *y*_0_, *z*_0_) = (0.4,0.5,0.5) for the bifurcation parameters: (a) *a* ∈ (0, 1) and (b) *c* ∈ (0, 1).

**Figure 10:** Time behaviors of state variable *x*(*t*) of commensurate FOCM (2) for different fractional orders and system parameters: (a) *a* = 0.1, (b) *a* = 0.50, (c) *b* = 0.1, (d) *b* = 0.53, (e) *c* = 0.1, and (f) *c* = 0.35.

The article "Chaos in Cancer Tumor Growth Model with Commensurate and Incommensurate Fractional-Order Derivatives" was published in 2022. Journal: Comput Math Methods Med.

**Figure 11:** Incommensurate FOCM (2) for *a* = 0.7455, *b* = 0.7367, *c* = 0.5619, and (*x*_0_, *y*_0_, *z*_0_) = (0.4,0.5,0.5). (a) Bifurcation diagrams for *q*_1_ ∈ (0.6,1), *q*_2_ = *q*_3_ = 1, *q*_2_ ∈ (0.6,1), *q*_1_ = *q*_3_ = 1, and *q*_3_ ∈ (0.6,1), *q*_1_ = *q*_2_ = 1 and (b) LLEs for *q*_1_ ∈ (0.86,1) and *q*_2_, *q*_3_ ∈ (0.85,1).

**Figure 12:** Time behaviors of the state variables: *x*(*t*), *y*(*t*), and *z*(*t*) (in red, blue, and green color, respectively) of the incommensurate FOCM along with the corresponding phase portraits in *x*-*y* plan when *a* = 0.7455, *b* = 0.7367, *c* = 0.5619, and (*x*_0_, *y*_0_, *z*_0_) = (0.4,0.5,0.5) for: (a) *q*_1_ = 0.999, *q*_2_ = *q*_3_ = 1, (b) *q*_2_ = 0.999, *q*_1_ = *q*_3_ = 1, and (c) *q*_3_ = 0.999, *q*_1_ = *q*_2_ = 1.

**Figure 13:** Bifurcation diagrams of the incommensurate FOCM (2) with *a* = 0.7455, *c* = 0.5619, and (*x*_0_, *y*_0_, *z*_0_) = (0.4,0.5,0.5) by varying parameter *b* ∈ (0.2,1) for: (a) *q*_1_ = 0.999, *q*_2_ = *q*_3_ = 1, (b) *q*_2_ = 0.999, *q*_1_ = *q*_3_ = 1, and (c) *q*_3_ = 0.999, *q*_1_ = *q*_2_ = 1.

**Figure 14:** Chaotic attractors of incommensurate FOCM in 3D projection with taking initial conditions (*x*_0_, *y*_0_, *z*_0_) = (0.4,0.5,0.5), fixing parameters *a* = 0.7455, *c* = 0.5619, and parameter *b* = 0.38 for: (a) *q*_1_ = 0.999, *q*_2_ = *q*_3_ = 1, (b) *q*_2_ = 0.999, *q*_1_ = *q*_3_ = 1, and (c) *q*_3_ = 0.999, *q*_1_ = *q*_2_ = 1.

**Figure 15:** Time behaviors of the state variable *x*(*t*) of incommensurate FOCM (2) for different fractional-orders and system parameters: (a) *b* = 0.1, (b) *b* = 0.50, (c) *b* = 0.1, (d) *b* = 0.5, (e) *b* = 0.1, and (f) *b* = 0.50.

## Data Availability

The data that support the findings of this study are available upon request.

## Appendix

### A. Basic Concepts

We state certain key preliminaries in regard with the noninteger calculus [21]:

Definition 1 A.1. The integral operator of fractional-order q in the sense of Riemann-Liouville of the function g ∈ C^m^(0, T] is outlined as

(A.1) $$\begin{array}{c} I^{q}g\left(t\right)=\frac{1}{\Gamma \left(q\right)}\int_{0}^{t}\frac{g\left(s\right)}{{\left(t-s\right)}^{\left(1-q\right)}}ds, \end{array}$$

where *q* > 0, *m* ∈ *ℕ*, and *T* > 0.

Definition 2 A.2. The differential operator of fractional-order q in the sense of Caputo of the function g ∈ C^m^(0, T] is outlined as

(A.2) $$\begin{array}{c} D^{q}g\left(t\right)=\left\{\begin{array}{cc} \frac{1}{\Gamma \left(m-q\right)}\int_{0}^{t}{\left(t-s\right)}^{m-q-1}g^{\left(m\right)}\left(s\right)ds, & q\in \left(m-1,m\right),\\ g^{\left(m\right)}\left(t\right), & q=m, \end{array}\right. \end{array}$$

where *q* ∈ [*m* − 1, *m*], *m* ∈ *ℕ* and *T* > 0.

The article "Chaos in Cancer Tumor Growth Model with Commensurate and Incommensurate Fractional-Order Derivatives" was published in 2022. Journal: Comput Math Methods Med.

### B. Numerical Method for Solving Fractional Differential Equations

To approximate the fractional-order dynamical system using the ABM and PECE numerical approximation method consider [22]

(B.1) $$\begin{array}{c} D^{q}x=f\left(t,x\right), \end{array}$$

where *q* is the fractional-order, 0 ≤ *t* ≤ *T* with initial values *x*^*k*^(0) = *x*_0_^*k*^ for *k* ∈ [0, *n* − 1]. Equation (B.1) can be solved using the Volterra integral equation (VIE) given by

(B.2) $$\begin{array}{c} x\left(t\right)=\overset{n-1}{\underset{k=0}{\sum }}x_{0}^{k}\frac{t^{k}}{k!}+\frac{1}{\Gamma \left(q\right)}\int_{0}^{t}\frac{f\left(\tau ,x\right)}{{\left(t-\tau \right)}^{1-q}}d\tau . \end{array}$$

The numerical approximation form of (B.2) can be defined as

(B.3) $$\begin{array}{c} x_{h}\left(t_{n+1}\right)=\overset{n-1}{\underset{k=0}{\sum }}x_{0}^{\left(k\right)}\frac{t_{n}^{k+1}}{k!}+\frac{h^{q}}{\Gamma \left(q+2\right)}f\left(t_{n+1},x_{h}^{p}\left(t_{n+1}\right)\right)+\frac{h^{q}}{\Gamma \left(q+2\right)}\sum a_{j,n+1}f\left(t_{n+1},x_{h}^{p}\left(t_{n+1}\right)\right), \end{array}$$

where

(B.4) $$\begin{array}{c} \left\{\begin{array}{c} a_{j,n+1}=\left\{\begin{array}{cc} n^{q+1}-\left(n-q\right){\left(n+q\right)}^{q+1}, & j=0,\\ -2{\left(n-j+1\right)}^{q+1}, & 1\leq j\leq n,\\ 1, & j=n+1, \end{array}\right.\\ x_{h}^{p}\left(t_{n+1}\right)=\overset{n-1}{\underset{k=0}{\sum }}x_{0}^{\left(k\right)}\frac{t_{n}^{k+1}}{k!}+\frac{h^{q}}{\Gamma \left(2\right)}\overset{n}{\underset{j=0}{\sum }}b_{j,n+1}\left(t_{j}x_{h}\left(t_{j}\right)\right),\\ b_{j,n+1}=\frac{h^{q}}{q}\left({\left(n-j+1\right)}^{q}-{\left(n-j\right)}^{q}\right), \end{array}\right. \end{array}$$

*h* = *T*/*N*, and *t*_*n*_ = *nh* with *h* ∈ [0, *N*]. The error for this method can be estimated as *e*_max_ = max|*x*(*t*_*j*_) − *x*_*h*_(*t*_*j*_)| = 0(*h*^*p*^), where *i* = 0, 1, ⋯, *N* and *p* = min(2, 1 + *q*).
